RETRACTED

# Environmental and Geographical (EG) Image Classification Using FLIM and CNN Algorithms

**DOI:** 10.1155/2022/4989248

**Published:** 2022-08-17

**Authors:** P. Ajay, B. Nagaraj, Ruihang Huang, M. S. Pradeep Raj, P. Ananthi

**Affiliations:** ^1^Faculty of Information and Communication Engineering, Anna University, Chennai, India; ^2^Department of Electronics and Communication Engineering, Rathinam Technical Campus, Coimbatore, India; ^3^Donghua University, Shanghai, China; ^4^Department of Artificial Intelligence and Data Science, Rathinam Technical Campus, Coimbatore, India

## Abstract

Intelligent machines have grown in importance in recent years in object recognition in terms of their ability to envision, comprehend, and reach decisions. There are a lot of complicated algorithms that accomplish AI utilities. In addition to their use in the medical industry, these methods of object recognition have a wide range of other fields, most notably industries, in which they can be applied. In contrast to the proposed calculation, the proposed calculation is less complex and more accurate under certain SNR conditions. In the deep nervous tissue fine-tuning discriminator, phantom highlights and binding highlights are separated as sources; modified direct components are used as neuronal activation abilities; and cross entropy is used as unfortunate abilities. Optimized recognition of profound nervous tissue builds profound and periodic nervous tissue for regulatory confirmation of the corresponding signal.

## 1. Introduction

Creating this double virtual representation of a particular world is the methodology of processing digital images. This two-dimensional interpretation is incredibly useful in numerous fields, including the health world, the automation industry, and robotics. This data is utilised in numerous fields with high efficiency including its malleability and adaptability [1]. This data is used to classify extraction of features, multiscale parameter estimation, pattern classification, and projection, among numerous other processes[2, 3]. Because it has undergone the process of object recognition, the human visual system is capable of recognising nearly all objects. Object recognition is a technique that recognises the primary properties of an object in order to comprehend it [4]. This method has two fundamental phases: extraction of features and pattern matching or categorization. The segmentation techniques are the most crucial and difficult elements of an image feature identification system [5, 6]. The properties of an attribute are used to extract its characteristics. These properties consist of an object's coordinates, ordinary elements, color preconceptions, area, background ratio, etc. Depending on the application being used, feature extraction methodologies can vary. In the preceding decades, algorithms including such subspaces strategies have played an essential role. These methods collect 2D data using both high- and low-resolution techniques. Fisher'slinear discriminate collects the above linear projection of the data using the linear discriminate. Fisher's linear discriminate extracts the linear forecast from spatial quality and performance data, which is utilised primarily in palm recognition applications. The eigenvalue detection approach, which is the basis of many algorithms such as ICA, computes a random sample from image components [5, 7]. This method is used in various image processing applications. Using the Gaussian phase of the data as the starting point, this algorithm extracts the same important features. ISO integrates one of the nonlinear size reduction techniques, nonlinear discretization, into the quasi-isometric elevated data points used as features. In this case, a simple geometry [8, 9] is estimated using the data manifold. PCA, also known as the main core component, is a proven method that uses the kernel method to increase the reliability of detection. This KPCA uses Hilbert spaces to determine the statistical data for multivariate regression of the dataset [10]. Applications including NLP have used the algorithm is known as semantic similarity analysis (LSA) [11] to process language. It utilises the terminology of the economic and financial hypothesis, whereby an SVD (Singular Value Decomposition) technique is utilised to decrease similar features between the various data articles [12]. The partial least square method is another time-tested data analysis technique. With the aid of a regression mechanism, this method estimates the data points. Multifactor Matrix Factorization is a method that is frequently employed for feature extraction [13, 14]. This process generates or recognises the characteristic combination of independent attributes, which ultimately results in the production of statistical features. It accomplishes this by employing a data mining strategy to process the functions. A semi-definite embedding (SDE) is a method used to perform a nonlinear dimensional reduction of a vector information source [15–17], and [18]. This method is utilised to reveal the data's maximum dimensions. Every one of these algorithms is fast, but they cannot do the following. Multiple object detection, optimised feature extraction, location identification, etc. In this paper, we introduce a method and a logical and systematic procedure that can be defined and compared to the corresponding scene to address the issues raised. This paper contributes to the FLIM automated system and an effective situation-context system.

RETRACTED

The following is a definition of object identification and multiobject acknowledgement in literary research and algorithmic study characteristics:

Ping Jiang and colleagues developed a vision-servoing algorithm for 3-D pattern classification and photo-shooting tracking. The algorithm records the image and determines IBVS. Data-driven unfalsified control is proposed to solve visual servoing problems. A recursive consensus mechanism manages feature modelling[19, 20]. Sebastien C. Wong and colleagues developed Responsive Manifestation Tracking. Without prior knowledge, this system tracks every object in a sequence or scenario. Due to dataset variations, trained detection systems may not encounter the items. However, this method will continue to search until the objects are recognised [21]. After detecting objects, a fast-learning picture classifier classifies them [24]. Strong echolocation algorithm for underwater computer vision was based on the sensor's angle of approach; this algorithm modifies the object's form. Detecting underwater objects is a computational challenge, as the system uses sonar simulator-based algorithms to propose techniques for detecting 3D objects and their poses. This algorithm solves the irregularity of 3D object detection. This algorithm can handle online and offline detections. Also, the two-step anticounterfeit filter produces more consistent 2D and 3D color pairs. After creating an online 2D to 3D object communication from the extracted features, a two-step fake communication filter is applied to the selected image. Each process step leading to pose evaluation and object transformation is completed. Also, the underwater fish detection framework was created to overcome the difficulty of detection. Reorganization requires a lot of data. To avoid framework limitations, emphasis, relaxed labeling to fit objects to unsupervised formation criteria, and classification decisions were used. The worldwide theory verification framework identifies overloaded 3D objects. The final stage of the 3D machine vision pipeline comes to a conclusion with theory confirmation to prevent false-hits. Whether these concepts are added depends on global or local features. Each theory is evaluated in this phase. There were issues with hypothesis confirmation, so the suggested technique replaces it. If the weak hypothesis is verified, it will correctly detect objects while remaining coherent. Additionally, they found that identifying organisms as well as objects with a restricted number of varieties, where their visual characteristics are captured by size, scale, and angle, is one of the most difficult challenges for computer vision. The algorithm worked in the previous variations, but still fails whenever the object rotates or moves too much. Living things can recognise uniform artifacts and animals. The feedforward construct stimulates the visual system to help the HMAX model recognise objects. Each stage models single cells for selectivity and complex cells for invariance. The HMAX model employs sparse coding, which eliminates sensitive features while improving classification. Atoms with high correlations balance the factors. Feature-Graph framework uses concurrently associated ideas to detect and model items. The proposed framework depicts artefacts as graphs with vertices and edges. Three-dimensional object observation is used in object modelling. The concurrent entity identifier and model-based problem require maximum likelihood estimation.

RETRACTED

## 2. System Overview

This section explains the environment identifier's architecture.  Figure 1 depicts the proposed research methodology. Most computer vision algorithms process nonlinear real-world data. Nonlinear data and scenarios are processed using ANN, Fuzzy Logic, and Neuro-Fuzzy methods. GA and PSO are used to find the best way to complete a task. Deep learning improved AI in fields like recognition and deep learning, sparking a technological revolution. This essay is about understanding one's natural surroundings (the situation of a place where computer vision is framed). This scenario calls for Section 4 deep learning.  Section 5 explains how to cluster.  Section 6 describes all processes internally. Last section Sections 7and 8 include findings, discussion, and a summary.

## 3. CNN for Environment Identifier

Both enviromental identifier procedures use CNNs. Object recognition uses R-CNN. This algorithm compares objectless. This convolutional network is an RPN. The system contains five sharable convolution layers, as per Zeiler and Fergus. Moving the object proposals window over convolutional feature maps determines the network's regions. This spatial window collects low-dimensional features for use by its sister layers. Classification and regression. Anchors were strategically placed to retrieve the most potential regional proposals. Each anchor's window size will be adjusted so that comprehensive data inquiries can be made. Consider this: Anchors have five windows. The size of the feature map determines the total number of windows used. It primarily generates a list of visible items. This list can be used variously. An object list helps identify the scene's main elements.

S–CNN does have five layers: an input, an outcome, and three hidden unit layers. A first multiple hidden layers activate convolution layers filtering and pooling. Scale or translation-invariant features are extracted after input via convolutional filtering and pooling. Classification is complete with the third hidden and output layers. Convolution layers filtering and pooling were used to analyse KPD (key point discriminators). Multiple objects in a scene are organised as a 2D set of data for the S-input CNN's layer, along with KPD generated from feature extraction, background object concentration, color density, and regional information. This guarantees data accuracy. This block uses filters to process visual data inputs. These filters process data. The second hidden layer's linearly concatenated features are then used to activate the third. The second hidden layer's projections were linearly concatenated. Activating neuronal circuits helped develop classification-based predictions. Using S–CNN to classify environmental features will help you reach your goal. The EG Identification classification will be decided after R-CNN and FLIM input. Training uses many identical samples as well as labels. These neutral connections are tested for analysis and performance.

RETRACTED

## 4. Fuzzy Local Information Means (FLIM) Algorithm

Traditional K-Means clustering uses vector quantization. In most cases, a recursive method chooses the cluster's centre by chance and then manipulates distance measurement. The cluster centre is determined by the previous iteration's mean. Each iteration performs this calculation. Recalculating clusters will continue until convergence is reached. The K centres' positions change with full convergence. What is happening is causing this. The traditional K-Means algorithm has three parts: (1) convergence function, (2) cluster centre recalculations, and (3) cluster bin.

(1) $$\begin{array}{c} C_{f}=\sum_{i=1}^{nc}\left(C_{c}i-NC_{c}i^{2}\right), \end{array}$$

(2) $$\begin{array}{c} NC_{c}i=\left(\frac{1}{n\text{d}c_{i}}\right)\sum_{j=1}^{n\;dc_{i}}Cbin_{i}, \end{array}$$

(3) $$\begin{array}{c} Cbin_{i}=Cbin_{i}|X_{S}i, \end{array}$$

(4) $$\begin{array}{c} X_{S}i=\lim_{j=1\text{ to }nx}x_{j}\text{if dist of }x_{j}\text{is}\min\text{ to }C_{C}i, \end{array}$$

(5) $$\begin{array}{c} \text{dist}=x_{j}-C_{c}i^{2}\left\{\frac{j=1\text{ to }nx}{i=1\text{ to }nc}\right\}. \end{array}$$

This function calculates cluster centre dissimilarity. It is possible to define stopping criteria and control recursive stages, but this depends on accuracy. This reflects the user's requested or available clusters. This section compares the current and future cluster centres. Based on the cluster bin mentioned earlier, the formula where and are equal determines the number of cluster bins. The number of clusters required is equal to the number of bins formed. The number of accessible data elements is equal to the number of points or elements that are the minimum distance apart.

RETRACTED

This method of evaluating data processing has the following limitations: (1) Linear. This means that the data in one cluster is not available in another cluster, but this is unlikely to be real-time. The K-means method can converge to the local minimum instead of the global minimum. The first random selection affects the final cluster despite the impact of the global minimum. (3) Minimal movement—during each iteration, adjustments to the cluster centres are kept to a minimum, which increases overall time complexity. This led to the creation of the fuzzy local information means (FLIM), which is be discussed as follows :

(6) $$\begin{array}{c} lin_{ji}=\frac{1}{\text{d}ij}{\left(Max\left(x\right)-C_{c}i\right)}^{f}. \end{array}$$

Equation (6) displays cluster-specific local information. This is determined using the inverse Euclidean distance of data and the centres of both clusters. This function solves the optimum solution problem and pushes cluster centres to reduce total convergence rate.

If yes, FLIM's membership function is the same as K-Mean's (equation (2)) which includes improving the push-in cluster centre selection parameter.

(7) $$\begin{array}{c} NC_{c}i=\left(\frac{1}{n\text{d}c_{i}}\right)\sum_{j=1}^{ndc_{i}}M^{f}i+lin_{ji}, \end{array}$$

(8) $$\begin{array}{c} M^{f}k=X_{s}k\forall W_{k}, \end{array}$$

Here, n and nc is the no. of clusters requested by user.

*W* is the weight assigned for each cluster group element to show the difference between one and another.

In addition to being the function that is used to compute it, *NC*_*c*_*i* is also the function that holds the clusters that have previously been grouped together based on the previous computation *C*_*c*_*i*. Equation (8). Additionally, the function is the one that takes into account the clusters *X*_*S*_*i* that have been grouped together based on the preceding computation. What sets FLIM apart from the competing approach *M*^*f*^*k* is its fuzzy character, which would not have been considered in the conventional K-means calculation The conventional approach did not involve the presence of this fuzzy quality. This includes cluster groups whose members may be in another cluster.

(9) $$\begin{array}{c} X_{S}k=\lim_{j=1\text{ to }nx}x_{j}\text{ if }d_{ij}\text{ of }x_{j}\text{is}\min\text{ to }C_{C}k,\\ d_{ij}=x_{j}-C_{c}i^{2}\left\{\begin{array}{c} j=1\text{ to }nx\\ i=1\text{ to }nc \end{array}\right\}. \end{array}$$

The data that was selected for each cluster can be found in equations (9) and (10) along with the distance measurement that was taken between the data elements and the group. This determined the degree to which the data elements matched the cluster. Following the selection of these data, data points containing people are given a high priority on the cluster, while quasi data sets are given a lower priority.

(10) $$\begin{array}{c} Obj_{f_{Iter}}=\sum_{i=1}^{nc}\sum_{j}^{nx}M^{f}id_{ij}+lin_{ji}. \end{array}$$

By identifying the objective function that is responsible for making this decision, the recursive process also determines the degree of convergence. Optimization problems use membership factors that actually act in addition to the knowledge parameters specific to the data provided when trying to determine when convergence occurs. As a result, the implementation of fuzzy k-means at work was completed successfully. The following Figure 2 shows a step-by-step breakdown of the process required to implement this algorithm:

- The necessary inputs for the operation are described in the beginning of the process. These factors include the required number of clusters, the direct scores, and the associated information that should be clustered together.
- For the first iteration of the process, the cluster centres will be chosen at random from among the data points. What determines the locations of these centres of the cluster is that once random cluster centres are selected from the random vector, it is used to compute the distance measurement techniques varying according to cluster accuracy requirements and cluster nature.
- When generating the membership data, we make use of both random clusters and clusters that were produced by earlier iterations of the algorithm. The priority of the cluster serves as the determinant for the fuzzy weights that are incorporated into the membership data. However, this could only be done once the consolidation state has been reached, as the membership function is the individual's soul output.
- We will check for convergence at the end of each iteration using the optimal solution besides calculating its significance using the formula. This will be done using the objective function:

(11) $$\begin{array}{c} Obj_{f_{Iter}}-Obj_{f_{Iter-1}}<Cgnc_{cri}, \end{array}$$

where *Cgnc*_*cri*_ is an application-specific user-defined convergence criteria.

  If convergence state is attained
  Intration stops and the final membership function
  Values will be taken as the final outcome
  else
  The recrusive process continues from step(b)

RETRACTED

## 5. Operation

Using FLIM and deep learning to analyse and classify location and scenario is a methodical process with many steps. This study aims to establish a system that really can understand its operating conditions and spot irregularities. To perform this operation, a wide range of important characteristics must be gathered from both the object learning organisation and the backstory learning organisation. Object developed the R-CNN deep learning algorithm. This algorithm lists objects using anchor sliding windows in various configurations. FLIM is used in background learning. This is for the background. A key Point after FLIM's equations separate the object and background is that the traditional classifications of the input scene are extracted in 2 dimensions for S-classification CNNs. CNNs determine if a scene depicts a place or a situation. This section explains each step in detail:

- Both online and offline cameras can enter photos into the system. A moving topic is occasionally captured in still photos and films. Motion blur and noise reduction need to be eliminated for approaches-based processing.
- The input stage has two parallel sections. Object learning and background learning. R-CNN will perform object detection and recognition according to Section 4. After obtaining features and learning, we classify the objects to find a list. The object list is used in the next sorting phase.
- A fast and efficient clustering approach is used. This clustering uses 2D input data to differentiate between foreground and background. FLIM will collect input data consistent with Section 5 clustering process. The 2D membership function will produce a segmented image as a result.
- To extract the history, we take the common provinces of all the segmented outcomes and ignore the background. We can then extract its background. The procedure for extracting KPD features will consider context.
- BG density, color density, region index, texture index and color density, are KPD's four stages.

The texture index extracts insightful qualities from an image's spatial regions. Gray level frequencies as well as intensities affect image contour. Statistical measurements of the image extract power, local fractal dimension, and increasing input group to form a dual feature configuration. Feature agreement. History image co-occurrence matrix generate statics.

(12) $$\begin{array}{c} \epsilon =\sum_{r}\sum_{c}C_{a}{\left(r,c\right)}^{2}, \end{array}$$

(13) $$\begin{array}{c} \varepsilon n_{p}=-\sum_{r}\sum_{c}C_{a}\left(r,c\right)log_{2}C_{a}\left(r,c\right), \end{array}$$

(14) $$\begin{array}{c} H_{ty}=\sum_{r}\sum_{c}\frac{C_{a}\left(r,c\right)}{1+\;\left|\;r-c\;\right|}. \end{array}$$

These statics were obtained by sliding and moving windows across the image sequence. As a result, the and size are still 3, 5, 7, etc.

RETRACTED

In addition to texture statistical data, an image's reference details must be evaluated to learn as much as possible about the scene. This is done to gather as much information as possible about the scene. Once object details can be seen, the background's probability distribution estimate must be derived.

(15) $$\begin{array}{c} \mu_{f}=\rho I_{f}+\left(1-\rho \right)\mu_{f-1},\\ \sigma_{f}^{2}=d^{2}\rho +\left(1-\rho \right)\sigma_{f-1}^{2}, \end{array}$$

where *d* is the distance between the image and the generated mean value. This gives the background variety. So it fits the space-time PDF.

Multilevels of color density. Histogram measurements show the ratio of color to pixels. Color segmentation separates the foreground and the color scheme. Once these features are established, two types of information about color density can be collected. Statistics on available colors and information on dominant colors. Otsu threshold extracts the characteristics of the area index. This step uses a histogram of parallel feature extractions and intergovernmental thresholds for background images. All layers from the facility and tissue pixels are extracted using edge detection. All KPD functions are collected in a two-dimensional structure using the R-List-CNN of the particles, and the S–CNN identifies the environment. FLIM and Learning Techniques are systematic classification processing algorithms.

### 5.1. Results and Discussion

In this chapter, the specifics of a dataset that was utilised for the research are investigated, along with the modelling process. This process includes Training and classification, as well as the specifications that were used for assessment and the metrics that were used for the performance review. The algorithmic components and stages of the recognition system are decided upon following the execution of a series of experiments and the subsequent analysis of the data obtained from those experiments. In order to train and test the DL algorithms, a large number of multiobject images from a variety of databases, such as the KITTI Vision and MOT Challenges database are the Benchmark Suite database, amongst others, are used. The MOT Challenges and the KITTI Vision Benchmark Suite are both included in these databases. The following four classifications can be used to classify the various pieces of equipment that were utilised in the experiment: I Performance in terms of the identification of a large number of objects, performance in terms of FLIM, and performance in terms of the identifier of the surrounding environment (iv) Tables (1), (2), and (3) present the findings of these studies in the order in which they were obtained (3). The S–CNN algorithm needs to consult a number of databases, including NORB, MNIST, SVHN, and CIFAR, in order to evaluate the performance of multiobject detection. This is done so that it can determine how effective the technique is. The conventional K-Means algorithm, the FCM algorithm, the FCM S1 method, the FCM S2 method, the EnFCM method, and the FLICM method are contrasted with the FLIM method. This is done with the goal of analysing how well it works in comparison to all these other algorithms and drawing conclusions based on those findings. The following are some of the inferences that can be made following the completion of this analysis.

RETRACTED

Using the test cases that are contained within a range of benchmark datasets allows for an accurate evaluation of the effectiveness of multi-object detection. This gives a balanced and truthful portrayal of the reality in which we actually live. In this part of the chapter, both the Miss Ratio and the False-Hit Ratio are calculated, and Table 1 contains the findings of both calculations. The ratio of genuinely correct data that was missed from recognition is referred to as the “miss ratio,” whereas the fraction of actually incorrect data that was classified as correct is referred to as the “false-hit ratio.” The varied findings that were acquired can be used to piece together a comprehensive image of the nature of the algorithm and its reaction for the distinct datasets.  Figure 3 can be gained from the results that were obtained.

The findings of the conflict between FLIM and many other clustering algorithms are shown in Table 2 and Figure 4, respectively. Developed here by analysing the conventional K-Means method, FCM (Fuzzy C Means) method, FCMS (FCM Spatial) method, EnFCM (enhanced fuzzy C means) method, FLICM (fuzzy local information C means) method [57]. Compared to the approach that was done the results make it very clear that these methods are specific to many different operations and categories. This conclusion can be drawn with absolute certainty. Some approaches cluster the information more quickly than the others, and some bunches are more effective than others at removing noise from the background than others. The FLIM algorithm is resilient enough to preserve a high level of segmentation accuracy; in particular, it addresses the problem of finding the global optimal solution. As a direct result of this, the period of hours and usually present is reduced, while the level of efficiency that was previously achieved is preserved.

Table 3 and Figure 5 show the results of the proposed algorithm's accuracy when it was simulated using a variety of databases. The recognition is carried out with the assistance of a convolutional neural network, thus these results are particularly relevant. The phase of training and testing needs to be carried out before an assessment of the network can be carried out. This will allow the network to be strengthened. The training phase for S–CNN is carried out during this stage of the procedure employing 600 photos collected from the MOT database along with its requisite classification targets [58].

RETRACTED

## 6. Conclusion

This article describes a technique for identifying and gaining knowledge of a location or scene for the purpose of conducting surveillance. Compiling recently developed and proposed algorithms and organizing them into a system was done with the intention of making this system more helpful. Finding those who are in need is made easier by combining FLIM, S–CNN, and FLIM. The performance of this system is up to all of the standards. In the not-too-distant future, this technique will be utilised for computer vision in robotics to make judgments and detect irregularities all around the planet. This has the potential to save thousands of lives all across the world. It has an accuracy rate of 89 percent on average when there is jitter and 94 percent when there is none [8, 22].

## Figures and Tables

**Figure 1:** Systematic Process view of the environment identifier.

**Figure 2:** A unified network of R-CNN.

**Figure 3:** Comparison of R-CNN.

**Figure 4:** The accuracy of a clustering algorithm in terms of background segmentation is compared.

**Figure 5:** Accuracy of the proposed environment classifier.

**Table 1:** Comparative analysis of R-CNN.

Databases	Miss (%)	False hit (%)
CIFAR	11.84	9.05
SVHN	13.53	7.91
MNIST	14.58	8.51
NORB	12.63	9.54
KITTI vision	12.91	7.67
MOT challenges	13.53	9.89

**Table 2:** A study evaluating the performance of several clustering algorithms with respect to background segmentation.

Image	K-Means	FCM_S	ENFCM	FLICM	M-FLMCM	FLIM
S-1	85.64	85.35	81.43	92.46	92.33	87.32
S-2	92.24	85.19	85.37	85.63	82.61	81.43
S-3	87.32	92.33	85.19	82.71	89.70	92.24
S-4	80.93	87.32	83.29	89.38	92.33	89.70
S-5	92.24	92.33	92.46	89.38	83.29	82.61
S-6	85.37	92.24	89.70	80.93	85.37	85.64
S-7	89.38	85.64	85.19	85.19	82.61	82.71
S-8	92.46	82.71	83.29	81.43	82.61	89.38
S-9	85.35	85.35	80.93	87.35	80.93	85.35
S-10	89.70	85.64	92.46	83.29	85.37	81.43

**Table 3:** Proposed environment classifier's accuracy.

Benchmark dataset	Training with jitter (%)	Validation with jitter (%)	Validation without jitter (%)
NORB	94.43	89.99	96.63
MNIST	97.34	94.92	90.4
SVHN	95.32	96.13	93.56
CIFAR	97.67	93.17	94.66
MOT CHALLENGES	93.21	94.47	90.19
KITTI VISION	89.95	90.30	96.89

RETRACTED

## Data Availability

The data used to support the findings of this study are available from the corresponding author upon request.
